# Feature Extraction and Small-Sample Learning of Dexmedetomidine for Neurosurgery on Postoperative Agitation in Patients with Craniocerebral Injury

**DOI:** 10.1155/2022/3699647

**Published:** 2022-03-15

**Authors:** Chuan Ding, Xiuhua Wang, Xiuqin Wang

**Affiliations:** ^1^Department of Anesthesiology, Shandong Cancer Hospital and Institute, Shandong First Medical University and Shandong Academy of Medical Sciences, Jinan, Shandong 250117, China; ^2^Department of Materials Chemistry, Anhui Normal University, Wuhu, Anhui 241002, China

## Abstract

*Objective*. To observe the controlled effect of dexmedetomidine for neurosurgery and the effect on postoperative cognitive function. The main task of this paper is to use data from a small sample. The proposed feature extraction algorithm based on the bilinear convolutional neurological network (BCNN) is based on a small sample of data. BCNN involves the simultaneous extraction of highly discriminative cross-sectional features from the input image using two parallel subnetworks. By optimizing the algorithm to minimize losses, the two subnetworks can be supervised by each other, improving the performance of the network and obtaining accurate recognition results without spending a lot of time adjusting parameters. The mean arterial pressure (MAP) and heart rate (HR) levels of cerebral oxygen metabolism were compared between the two groups before (T0), after (T1), immediately after (T2), and after intubation (T3). In the observation group, MAP and HR values at T3, arterial-internal jugular vein bulb oxygen difference [*D*(*a* − *jv*)*O*_2_] at T1, T2, and T3, cerebral oxygen uptake (CEO_2_) levels, and postawakening agitation scores were lower than those of the control group during the same period (*P* < 0.05).

## 1. Introduction

Craniocerebral injury in surgery is more traumatic and patients suffer from nervousness and fear, which require appropriate anaesthetic hypnosis to reduce the occurrence of stress reactions and improve surgical safety. Postoperative extraction, aspiration, and postoperative pain stimulation can lead to excitation of the sympathetic-adrenergic system, increased blood pressure levels, increased heart rate, and even cardiovascular and cerebrovascular accidents [1]. Dexmedetomidine is highly selective for *α*_2_ receptors, with an affinity more than 1,600 times that of *α*_1_ receptors, inhibits norepinephrine release [2], reduces postsynaptic membrane excitability, has a low preoperative aerodynamic impact, has no respiratory depressant effect, effectively inhibits sympathetic excitation, lowers catechol levels, and reduces the stress response. When combined with opinions, it can prolong the duration of opiate analgesia and enhance the sedative effect with significant effect [3].

Craniocerebral injury is a difficult procedure as the vertebral body and the surrounding tissues are rich in blood vessels and the operation site is deep, making it difficult to stop bleeding [4]. Patients undergoing craniocerebral injury are mostly middle-aged and elderly, mostly combined with underlying diseases, so maintaining the hemodynamic stability of patients is of positive significance to improve the safety of surgery [5]. Dexmedetomidine is a new highly selective *α*_2_-adrenergic agonist that can reduce the stress response during surgery and maintain aerodynamic stability [6]. This study will look at the effect of dexmedetomidine in controlled hypotension during craniocerebral injury and its effect on patients' postoperative cognitive function.

Under normal conditions, cerebral oxygen metabolic rate changes in synchrony with cerebral blood flow. When the cerebral oxygen metabolic rate increases, the cerebral vasculature also strengthens and automatically dilates, resulting in elevated cerebral blood flow, which can cause secondary brain damage to occur when the cerebral oxygen supply and demand are in an imbalance [7, 8]. In this study, we compared and analysed the differences in postoperative cognitive function between the two groups, and the results showed that cognitive function in the observation group was higher than that in the control group within a short period of time after surgery, which is consistent with the findings of Gunduz et al. [9], indicating that dexmedetomidine is beneficial to the recovery of cognitive function after anaesthesia. This may be due to the cerebral protective effect of dexmedetomidine, which reduces the cerebral oxygen metabolism rate, increases the superoxide dismutase content, and antagonises the brain damage caused by the anaesthetic.

In conclusion, dexmedetomidine is safe and effective for controlled hypotension in craniocerebral injury, effectively inhibiting cardiovascular responses during tracheal intubation, reducing the patient's preoperative cerebral metabolism level, and improving postoperative cognitive function.

## 2. Knowledge Background

### 2.1. Restlessness and Impact

Song et al. [10] define agitation as the hyperexcitability of the patient during the awakening period after the application of ether, cyclopropane, or ketamine anaesthesia, which is mainly manifested by unconscious movements of the limbs, uncontrollable crying, irrational speech, excitable agitation, and disorientation.

The causes of agitation are multiple and include surgical-related factors (postoperative incision pain and prolonged passive position), anaesthetic factors (partial anaesthetic drugs and residual effects of inotropic drugs), and various adverse stimuli (catheter and tracheal tube stimulation) [11]. However, it is still not possible to explain the exact mechanism by which all postoperative agitation occurs. Some scholars believe that it may be related to the different degrees of suppression of the central nervous system by anaesthetic drugs; such patients may have recovered consciousness during the awakening period of general anaesthesia, but due to the residual effects of some anaesthetic drugs, the patient's cerebral cortex is still suppressed, while their subcutaneous central functions have been restored. This inconsistent neurological state results in a lack of functional integrity of the brain, which ultimately leads to a state of central nervous system hyperexcitability [12]. This lack of functional integrity can take many forms, for example, after awakening from anaesthesia, the patient is generally quiet and drowsy, with a small number of patients having mild disorientation and a gradual normalisation of the functional brain response from blurred or sluggish, but a few of these susceptible patients can be agitated (reflexively antagonised) by any adverse stimulus (pain, distress, or discomfort) during the period of blurred or sluggish functional brain response [13].

### 2.2. Dexmedetomidine

*a*_2_ adrenoceptor (*a*_2_-AR) agonists are favoured by anaesthetists because of their unique mechanism of action in anaesthesia and the fact that they do not inhibit breathing. Dexmedetomidine (Dex) is a relatively recently discovered and used *a*_2_ adrenoceptor agonist, which was first used in the USA in 1999 for short duration (<24 h) sedation of ICU patients; it has since been used in a wide range of clinical applications due to its unique pharmacological properties [14]. DEX inhibits the release of norepinephrine from neurons by making brainstem pontine, calms the brain, and resists anxiety. Its unique feature is to keep the brain awake in the case of hypoxia. This advantage makes Dex unique in the type of surgery that requires intraoperative patient cooperation [15].

In the perioperative period, many patients have an excessive stress response due to fear of anaesthesia and surgery, resulting in excitation of the sympathetic nervous system and increased release of catecholamines, which is reflected in circulatory fluctuations such as increased heart rate and blood pressure [16]. Dex significantly inhibits sympathetic hyperexcitability and the release of noradrenaline from neuronal endings, improving perioperative blood flow stability and thereby reducing the risk of perioperative myocardial ischemia [17].

## 3. Bilinear Convolutional Neural Network (BCNN)

The main task of this paper is to identify the craniocerebral injury of dextromethorphan. Our proposed BCNN structure is shown in Figure 1 [19]. Its innovation lies in (1) using two parallel subnetworks to simultaneously extract highly discriminative cross-sectional features from the input image; (2) fusing the extracted features to obtain fine features that help in recognition; and (3) minimizing losses through an optimization algorithm; the two subnetworks can supervise each other to improve the performance of the network and obtain accurate recognition results without spending a lot of time to adjust the parameters. The following will introduce the method of this paper in detail at network initialization, data acquisition and preprocessing, BCNN network design, etc.

### 3.1. Network Initialization

Network initialization has a significant impact on training, and poor initialization tends to trap the neural network in a gradient-depletion trap. Aryan et al. [7] pointed out that low-level CNNs learn features similar to the edge portion of the mask obtained by Gabor kernel filtering, and as depth grows, the CNN gradually learns distinctive features of the object; Therefore, many researchers have tried to fine-tune the parameters of the classification layer of the model to cope with different task scenarios using a migration learning-based training strategy. For the case of this study, which has a small sample of labelled dextromethorphan surgery data and is prone to overfitting in training, a migration learning strategy was adopted to initialize the subnetwork of the BCNN model using the ImageNet pretraining model, while the remaining parameters were initialized using Kaiming [21] initialization. The Kaiming initialization makes the output in training closer to the Gaussian distribution, which is conducive to the convergence of the network. The learning rate is set to 0.1 for the migration learning parameter layer and 1 for the Kaiming initialization parameter layer and decreases as the number of model iterations increases to provide a fine-tuning effect. This strategy allows the network model to maximize the learning of the distribution of the target data.

### 3.2. BCNNs

In the BCNN dextromethorphan surgery recognition algorithm constructed in this paper, the feature extraction part consists of two parallel CNN subnetworks, using ResNet and SqueezeNet as the backbone of the subnetworks, referred to as BCNN-R and BCNN-S in the following. *β*=(*F*(*A*)*F*(*B*), *P*, *C*) represents the whole model, where F denotes the feature extraction layer of the network, F(A) and F(B) denote the features extracted from the two subnetworks, respectively, P denotes the outer product pooling function, and C is the classification function. The function of the feature extraction layer F is to map a point *l* on the input image *L* to a *J* × *M* dimensional feature, which is pooled by the P function given by equation (1), and the classification function C outputs the identified types using the softmax function in equation (2), where *O*_*i*_ is the output for class *i*.

(1) $$\begin{array}{c} \left(l,\text{L},F\left(A\right),F\left(B\right)\right)=F\left(A\right){\left(l,L\right)}^{\text{T}}F\left(B\right)\left(l,\text{L}\right), \end{array}$$

(2) $$\begin{array}{c} C_{i}=\frac{\exp\left(O_{i}\right)}{\sum_{i}^{c}\exp\left(O_{i}\right)}. \end{array}$$

BCNN-S chose SqueezeNet [22] as the backbone network, mainly using the Fire module, which consists of two parts: compression and extension. The compression module fuses features of multiple dimensions into fewer dimensions, firstly convoy the input image using 3 × 3 convolution kernels to obtain a feature map with a higher number of channels and then convoying the feature map of the previous layer using fewer 1 × 1 convolution kernels to integrate features across channels to achieve the goal of reducing the number of feature dimensions. The extension module adopts a design similar to that of the Inception network [23], extending from the width of the network, using 1 × 1 and 3 × 3 convolution kernels to convolve the obtained feature maps in cascade, increasing the linear representation of the model, and improving the generalisation capability. The structure of the Fire module is shown in Figure 2.

In target recognition tasks, the only commonly used classification model is the single-branch network, consisting of a convolutional layer, a pooling layer, and a fully connected layer. The fusion of F(A) and F(B) yields a bilinear feature *X*=**F**(*A*)^T^**F**(*B*) of size *M* × *M*, transforming *X* into a bilinear vector of *M*_2_ × 1 for classification using linear layers. Intuitively, the bilinear form allows the features *F*(*A*) and *F*(*B*) to be constrained to each other and the outer product can be calculated for all forms of their combination, similar to the expansion of the perfect square formula. The feature fusion formula is shown in the following equation:

(3) $$\begin{array}{c} F{\left(A\right)}^{\text{T}}F\left(B\right)=\left(\begin{array}{c} a_{1}^{\text{T}}\\ \vdots \\ a_{m}^{\text{T}} \end{array}\right)\left(\begin{array}{ccc} b_{1} & \cdots & b_{m} \end{array}\right). \end{array}$$

As the convolutional neural network is end-to-end, i.e., the input is the original data and the output is the prediction, the training can be optimized using the backpropagation algorithm. Let d*ℓ*/d*x* be the gradient of the loss function with respect to the input *x*. Then, the gradient is chained to *F*(*A*) and *F*(*B*), respectively, and the gradient is shown in the following equation:

(4) $$\begin{array}{c} \frac{\text{d}\ell }{\text{d}A}=F\left(B\right){\left(\frac{\text{d}\ell }{\text{d}x}\right)}^{\text{T}},\frac{\text{d}\ell }{\text{d}B}\\ =F\left(A\right)\frac{\text{d}\ell }{\text{d}x}. \end{array}$$

From equation (4), we can see that A and B influence each other's gradients, i.e., they play a supervisory role, so the model can fully learn the subtle differences between the different categories to avoid overfitting, and even without deliberately adjusting the model hypermastigote, we can get better recognition results [24, 25].

## 4. Case Studies

### 4.1. Materials

The study was approved by the hospital ethics committee. Patients undergoing craniocerebral injury in our hospital from August 2016 to October 2018 were selected. Inclusion criteria were as follows: (1) patients with lumbar disc herniation or lumbar spine fracture who underwent elective surgical treatment in our hospital; (2) age 18–80 years; (3) American Society of Anesthesiologists (ASA) classification: grade I-II; (4) complete clinical data. Exclusion criteria were as follows: (1) combined with cranial trauma or severe central nervous system injury; (2) combined with hypertension, coronary artery disease, cardiac insufficiency, or severe cardiac arrhythmia; (3) combined with cardiac, hepatic, or renal dysfunction; (4) combined with coagulation or immune dysfunction; (5) presence of opium addiction, alcoholism, or drug abuse; (5) long-term use of immunosuppressive drugs; (6) combined with acid-base or electrolyte disorders; and (7) other internal endocrine disorders such as acid-base balance or electrolyte disorders. The 50 cases in the observation group were missing 2 cases due to follow-up, and a total of 48 cases were included, including 30 males and 28 females (age 35–77 years, mean (58.9 ± 5.9) years; body mass 47–81 kg, mean (61.9 ± 3.2) kg); 3 cases were illiterate, 8 cases were primary school students, and 37 cases were junior high school students or above; ASA classification: 29 cases of grade I and 19 cases of grade II. In the control group, there were 50 cases and 4 cases were missing from the follow-up, and a total of 46 cases were included, including 30 males and 16 females (age ranged from 37 to 78 years, mean (58.9 ± 5.8) years; body mass ranged from 48 to 80 kg, mean (61.8 ± 3.2) kg); 5 cases were illiterate, 9 cases were in primary school, and 32 cases were in junior high school or above; ASA classification: 25 cases in class I and 21 cases in class II. There was no statistically significant difference between the above general information of the two groups (*P* > 0.05) [26].

## 5. Results

The differences in HR and MAP values at T0, T1, and T2 between the two groups were not statistically significant (*P* > 0.05). The HR and MAP values at T3 in the observation group were lower than those in the control group (*P* < 0.05) (see Table 1).

The differences in CE *O*_2_ and *D*(*a* − *jv*)*O*_2_ levels between the two groups at T0 were not statistically significant (*P* > 0.05), while CE *O*_2_ and *D*(*a* − *jv*)*O*_2_ levels at T1 and T2 were higher than those at T0 in the same group (*P* < 0.05)*O*_2_, *D*(*a* − *jv*)*O*_2_ (see Table 2).

T4, T5, and T6 were higher in the observation group than those in the control group (*P* < 0.05) (see Table 3).

The observation group had longer extubation and awakening times than the control group; the controlled hypotension time was shorter than that of the control group, and the postawakening agitation score was lower than that of the control group (*P* < 0.05) (see Table 4).

The difference in the occurrence of adverse reactions between the two groups was not statistically significant (*P* > 0.05) (see Table 5).

## 6. Postoperative Agitation Effect

There was no statistically significant difference in the time to recovery of breathing, time to awakening, and time to extubation between the two groups (*P* > 0.05) (see Table 6).

The HR and MAP of group C were significantly higher than those of group D at all time points within 60 min after intubation, which was statistically different (*P* < 0.05). The differences in HR and MAP at 120 min after intubation were not statistically significant between the two groups (*P* > 0.05) (see Figures 3 and 4).

The Riker sedation and agitation scores at 60 min after extubation were statistically significantly higher in group C than in group D (*P* < 0.05). There was no statistically significant difference in the Riker sedation agitation scores at 120 min after extubation (*P* > 0.05) (see Figure 5).

The degree of agitation from the end of surgery to 120 min after extubation was higher in group C than in group D. The incidence of agitation was significantly higher in group D. There was a statistical difference (*P* < 0.05) (see Table 7).

The Ramsay sedation scores of patients in group C were statistically significantly lower than those of group *D* at all points within 60 min after extubation (*P* < 0.05). There was no statistically significant difference in Ramsay sedation scores between the two groups at 120 min after extubation (*P* > 0.05) (see Figure 6).

The results should be related to the sedative effect of dexmedetomidine, and dexmedetomidine can also reduce patients' pain and relieve the negative emotion of nervousness and anxiety and fear to a certain extent while sedating them, thus reducing the occurrence of agitation [2]. This study also showed the Ramsay sedation scores at the moment of awakening and the moment of exultation.

In addition, oversedation is a possible risk after dexmedetomidine application. Ramsay sedation score is commonly used by clinicians and anaesthetists to analyse the level of sedation of patients. In this study, the Ramsay sedation score of both groups was below 4, although the score of group D was higher than that of group C, suggesting that dexmedetomidine infusion had a good sedative effect and that no oversedation occurred in this study.

In conclusion, dexmedetomidine hydrochloride is an adjunct to general anaesthesia with certain advantages. The treatment protocol of a preinduction loading dose of 1 *µ*g/kg (10 min) and a maintenance dose of 0.5 *µ*g/kg-h continuous infusion is effective and safe to use, resulting in smoother hemodynamics during recovery from general anaesthesia after craniotomy in patients with, less postoperative agitation, and less interpretative anaesthetic. It is safe to use and results in more stable hemodynamics, less postoperative agitation, less introspective anaesthesia, and a lower incidence of postoperative chills and delirium.

## 7. Conclusions

The proposed feature extraction algorithm based on a bilinear convolutional neural network consists of simultaneous extraction of highly discriminative cross-sectional features from the input image using two parallel subnetworks. Dexmedetomidine can be safely used for controlled hypotension in craniocerebral injury to reduce preoperative cerebral metabolism and improve postoperative cognitive function.

## Figures and Tables

**Figure 1:** BCNN structure.

**Figure 2:** Structure of the Fire module.

**Figure 3:** HR.

**Figure 4:** MAP.

**Figure 5:** Riker score.

**Figure 6:** Ramsay score.

**Table 1:** Comparison of mean arterial pressure and heart rate between the two groups at different time points.

Group	*n*	HR (times/min)				MAP (mmHg)			
		T0	T1	T2	T3	T0	T1	T2	T3
Observation group	48	74.1 ± 7.1	62.3 ± 6.9	65.6 ± 3.4	73.6 ± 9.3	93.9 ± 9.1	93.9 ± 9.1	93.9 ± 9.1	93.9 ± 9.1
Control group	46	74.7 ± 8.0	63.1 ± 7.9	66.4 ± 5.2	78.3 ± 9.8	94.3 ± 7.3	65.5 ± 7.4	66.9 ± 7.7	99.9 ± 7.5

**Table 2:** Comparison of cerebral oxygen metabolism levels between the 3 groups of patients at different time points ($\bar{x}\pm s$).

Group	n	CEO_2_ (%)				*D*(*a* − *jv*)*O*_2_ (Ml/dL)			
		T0	T1	T2	T3	T0	T1	T2	T3
Observation group	46	27.5 ± 6.5	31.3 ± 5.2	31.1 ± 3.9	28.1 ± 6.1	4.1 ± 0.8	4.0 ± 1.1	4.1 ± 1.1	4.4 ± 1.1
Control group	48	26.9 ± 6.3	39.5 ± 5.1	37.0 ± 5.2	35.4 ± 5.3	4.1±1.5	6.4 ± 1.0	5.7 ± 0.9	5.9 ± 1.2

**Table 3:** Comparison of postoperative cognitive function between the two groups.

Group	n	T0	T4	T5	T6	T7
Observation group	48	28.7 ± 1.1	25.5 ± 0.9	26.5 ± 0.3	27.9 ± 0.8	28.8 ± 0.9
Control group	46	24.2 ± 0.8	25.5 ± 0.4	26.2 ± 0.8	28.8 ± 2.1	28.7 ± 0.8

**Table 4:** Comparison of the quality of awakening between the two groups.

Group	n	Controlled depressurization time (min)	Extubation time (min)	Waking time (min)	Agitation score (point)
Observation group	48	72.4 ± 9.8	18.1 ± 3.0	17.8 ± 2.2	1.6 ± 0.4
Control group	46	79.8 ± 9.1	15.1 ± 3.3	14.7 ± 2.1	2.3 ± 0.4

**Table 5:** Comparison of the occurrence of adverse reactions in the two groups (cases).

Group	n	Nausea	Vomit	Drowsiness	Total
Observation group	48	2	1	2	5
Control group	46	1	2	1	4

**Table 6:** Recovery of basic postoperative signs (min, $\bar{x}\pm s$).

Group	Number of cases	Respiratory recovery time	Wake up time	Extubation time
Group C	20	4.3 ± 2.3	5.5 ± 2.9	9.1 ± 3.2
Group D	20	4.2 ± 2.1	5.3 ± 3.1	9.2 ± 3.1

**Table 7:** Occurrence of postoperative agitation in both groups (cases; ﹪, $\bar{x}\pm s$).

Group	Number of cases	Each agitation grade count					Incidence of agitation (%)
		3 points	4 points	5 points	6 points	7 points	
Group C	20	0	4	6	7	3	80
Group D	20	2	13	4	1	0	25

## Data Availability

The data underlying the results presented in the study are available within the article.
